# Towards Energy-Efficient and Delay-Optimized Opportunistic Routing in Underwater Acoustic Sensor Networks for IoUT Platforms: An Overview and New Suggestions

**DOI:** 10.1155/2022/7061617

**Published:** 2022-03-17

**Authors:** Varun G. Menon, Divya Midhunchakkaravarthy, Aaromal Sujith, Sonali John, Xingwang Li, Mohammad R. Khosravi

**Affiliations:** ^1^Department of Computer Science and Engineering, Lincoln University College, Petaling Jaya 47301, Malaysia; ^2^Department of Computer Science and Engineering, SCMS School of Engineering and Technology, Ernakulam 683576, India; ^3^Center of Postgraduate Studies, Lincoln University College, Petaling Jaya 47301, Malaysia; ^4^School of Physics and Electronic Information Engineering, Henan Polytechnic University, Jiaozuo 454000, China; ^5^Department of Computer Engineering, Persian Gulf University, Bushehr, Iran

## Abstract

In underwater acoustic sensor networks (UASNs), the reliable transfer of data from the source nodes located underwater to the destination nodes at the surface through the network of intermediate nodes is a significant challenge due to various unique characteristics of UASN such as continuous mobility of sensor nodes, increased propagation delay, restriction in energy, and heightened interference. Recently, the location-based opportunistic routing protocols seem to show potential by providing commendable quality of service (QoS) in the underwater environment. This study initially reviews all the latest location-based opportunistic routing protocols proposed for UASNs and discusses its possible limitations and challenges. Most of the existing works focus either on improving the QoS or on energy efficiency, and the few hybrid protocols that focus on both parameters are too complex with increased overhead and lack techniques to overcome communication voids. Further, this study proposes and discusses an easy-to-implement energy-efficient location-based opportunistic routing protocol (EELORP) that can work efficiently for various applications of UASN-assisted Internet of Underwater Things (IoUTs) platforms with reduced delay. We simulate the protocol in Aqua-Sim, and the results obtained show better performance than existing protocols in terms of QoS and energy efficiency.

## 1. Introduction

The genesis of life on Earth had its inception on water, from which it went on to conquer varied frontiers. With the advent of the latest technologies, today's world is more connected than ever before, but ironically the blue planet still lacks efficient underwater connectivity. Underwater acoustic sensor networks (UASNs) [1–3] made their way into the limelight of research quite recently; its pivot objectives deal with an array of versatile interests from oceanographic studies dealing with marine geology, marine ecology, and physical and chemical oceanography. Another significant application is resource extraction, which mainly concerns harnessing abundant rare-earth minerals, petroleum, and natural gas under the sea bed, calamity prevention, deep-sea climate monitoring, and protection, surveillance, and reconnaissance of strategic waters by naval forces around the globe. Conventional methods used for undertaking these tasks mentioned above require humans to physically dive into the ocean's depths or rely on remotely operated underwater vehicles (ROUVs). After the data collection process gets over, these units resurface to provide the output. The data acquired always fell short of fulfilling its objectives as there were problems like the lack of accurate real-time data, stringent storage constraints, inability in handling mobility, and capability to withstand underwater pressure.

UASNs have cell-powered sensor nodes deployed throughout the ocean bed that interact with each other and with the sonobuoys located at the surface to suffice these objectives. Their presence ensures effective communication with the sensor nodes (real time), and they are also the first responders to notify the base station if any nodes fail. Besides all these conspicuous merits, they have been used in underwater acoustic research and antisubmarine warfare for a long time, reflecting its practicality as the UASN's function under tight frequency limitations. Numerous unique features of the underwater environment make the deployment and use of UASN quite a challenging task [4–7]. Underwater conditions are different from the situations on land where the communication takes place with radio frequency (RF) aid. Unfortunately, the underwater environment consumes the energy of the RF waves and renders itself impractical. The mobility of underwater sensors with the ocean currents is another major challenge. To get better off from the challenging underwater situations, UASNs communicate using acoustic waves [8–10]. Underwater acoustic waves typically operate in the frequency range of 10 Hz to 1 MHz. The delay of propagation accompanies this slender range, but it seems to be the only viable choice forward on modicum energy store. UASNs make another edge by facilitating interfaces to communicate with autonomous underwater vehicles (AUVs) remotely. This feature will exponentially increase the range of AUV control, and this merit will also help us perceive the underwater world for research with an added advantage of burgeoning the amount of ocean monitored by human beings, which currently accounts for only 5%. Routing of data packets right from the sensor nodes to the sonobuoys and to surface stations is one of the most challenging issues faced in UASNs, primarily due to the rapid energy drainage, limited bandwidth, significantly high latency, and reduced reliability [11–17].  Figure 1 presents a sample application scenario of UASNs.

Terrestrial wireless sensor networks (TWSNs) have a conventional set of routing protocols that ensure good network performance. TWSNs at no point of operation face interruptions similar to ocean currents. Doppler spreading, interim path loss, and link quality loss create numerous challenges for routing in underwater environments. In a nutshell, the quality of service (QoS) and energy constraints of UASNs inextricably impede it from resorting to routing protocols of TWSNs. Majority of all the routing protocols proposed for TWSNs, thus proving to be powerless when it comes to UASNs. Numerous unconventional routing protocols were put forth in recent years for UASNs, and each focused-on energy efficiency, thus improving various QoS parameters like throughput, latency, load balancing, and robustness. Some of these protocols have already been tested for research, military applications, and catastrophe prediction. The selection of an appropriate routing protocol is significant as it is answerable for the reliable deliverance of data packets to the destination.

Table 1 presents the variations between the terrestrial wireless sensor networks (TWSNs) and underwater acoustic sensor networks (UASNs). Routing protocols in UASN face numerous design challenges. The weightage given to path selection accounts for the various problems that have to be confronted in the underwater environment, such as marine aquatic life, acoustic disturbances, propagation delay, and seismic shadow zones. Many new routing protocols are proposed to tackle these dilemmas; however, most of them lack the description of appropriate routing strategies. Routing strategies advocate the parameters, which will be extensively useful for researchers and other professionals to calibrate the effectiveness of algorithms used in UASNs to develop a strategy to tackle limitations like high propagation delay and energy usage. Picking the suitable scheme ensures engineers achieve desired productivity in applications. The routing protocols for UAWNs are mainly classified into location-based protocols and location-free protocols. The location-based protocols instrument the use of the information contained in the sensor nodes that are mostly two/three-dimensional position coordinates. In contrast, location-free/depth-based protocols depend mainly on pressure information present in sensor nodes. Most of the earlier conventional protocols proposed for UASNs selects the best path for sending data beforehand without considering the dynamic nature of the network environment. This negligence of the traditional routing protocols tends to compromise the use of the widespread resources in the network and can also pave the way to network failure. When setbacks like these started to portray, routing in UAWNs seems like an insurmountable dilemma, and the concept of opportunistic routing protocol (ORP) was then proposed [18–20]. This traction appeared due to various contributing factors like the increased need for extended capacity and expectation of top-notch QoS. The basic idea behind ORP turns the table on the demerit of unreliable transmission, that is, the undesired broadcast nature exhibited by the unreliable transmission is exploited here instead of selecting the nodes beforehand. The selection of nodes in ORP happens on the go. Numerous neighboring nodes (candidate set) receive the broadcasted message. The candidates belonging to the candidate set are sorted according to the metrics and prioritized based on the probability of becoming the next-hop forwarder. The candidate with the highest priority is given the ability to forward the data packets while others discard the packets. This is known as candidate coordination. Opportunistic routing protocols have proved their robustness and adaptability to uncertain conditions by showing their significant presence in many essential fields like oil/gas pipelines, power grids, and management of metro/railroads. Currently, the advancements closely related to ORP have not yet reached their pinnacle as many problems are yet to be solved. However, the prime intention that sleeps behind it is being the ability to make a set of independently weak nodes emerge together as a virtually robust set of links. Thus, ensuring reliability which in turn plummets the retransmission rates and chop down the energy consumption of UAWNs. All of these pros and cons will be thoroughly surveyed in this study.

The major contributions of the work are highlighted as follows:

- We review all the major location-based opportunistic protocols proposed for routing data packets in underwater acoustic sensor networks over these years. Numerous energy-based, QoS-based, and hybrid location-based opportunistic routing protocols have been proposed in 2019, 2020, and 2021, and they promise to provide much better performance to various real-time applications deployed in UASNs. Very few works have provided reviews on these latest protocols, and we initially tried to address this research gap. We analyze and present a brief description of their working mechanism and highlight their issues and challenges. These issues can be taken up in the future for further improvement in the design of routing protocols in UASN.
- From the review of the latest protocols, it is observed that increased delay and energy drainage are the two significant areas of concern that need further solutions. We then tried to model an easy-to-implement routing protocol that can guarantee energy efficiency with reduced delay to various applications deployed in UASNs.

The rest of the study is organized as follows: in Section 2, various applications using underwater acoustic sensor networks are discussed. The fundamental principles of opportunistic routing are explained in Section 3. Energy-based, QoS-based, and hybrid location-based protocols are discussed in Section 4. The proposed energy-efficient and delay optimized protocol is discussed in detail in Section 5. The future research directions are discussed in Section 6, and the study concludes in the next section.

## 2. Underwater Acoustic Sensor Networks

The planet we dwell upon is covered approximately with 71% of water. Under this blue element, lies countless untapped resources that will enable human society to advance in countless ways. In order to consolidate this final frontier, underwater wireless sensor networks prove to be the need of the hour. The underwater wireless sensor network (UASN) is the collection of self-driven sensor nodes and autonomous vehicles connected underwater to perform different collective tasks based on user applications. The sensor nodes can occupy different depth locations that will permit us to spread our reach even to the ocean's deepest places. The self-driven sensor nodes will collect and transfer the sensed data to the target destination using acoustic signals. The attractive applications of UASNs comprise real-time surveillance, disaster prevention, navigation assistance, water quality determination, industrial organization, fish tillage, underwater exploration, and pollution tracking. Almost each of these applications of UASN demands sensor nodes to transfer sensed data timely and precisely through the source node present underwater towards the destination node on the surface with the help of intermediate nodes in the network. However, due to the dynamic nature of UASNs, continuous node mobility, communication voids, and limited battery storage often lead to degraded network performance. In this complicated underwater environment, how to route data packets promptly and effectively even with the presence of a communication void is the most challenging research question.

### 2.1. Challenges in UASNs

This section presents an overview of various challenges in underwater acoustic sensor networks.

#### 2.1.1. Acoustic Communication

The terrestrial networks depend on RF waves to execute communication. Whereas the underwater environment is highly unpredictable, and RF waves are unfortunately absorbed. Additionally, a high amount of attenuation paves the way to energy loss; hence, RF waves are not an option to be considered. Optical waves cannot be regarded as a choice because the mobility of the nodes is unable to guarantee accuracy. The only viable option in this scenario is acoustic waves. Many other flaws are associated with the usage, but a suitable routing protocol is expected to sort out the dilemma.

#### 2.1.2. High Mobility

The underwater sensor nodes are constantly on the move. These movements are caused by ocean currents which arise due to wind, breaking waves, temperature, and salinity variations. For efficient data gathering, the movement of these nodes is vital and indispensable. However, in reality, this high mobility induces the formation of curves to the acoustic waves, which triggers the emergence of zones that makes some of the sensor nodes in the network unable to participate in data transfer, which brings forth performance issues to the network.

#### 2.1.3. Underwater Noise and Interference

The ocean is packed with a lot of noises and interferences that arise from varied sources. Some of the underwater noises are caused by breaking waves, rain, and marine life. However, various sources are man-made like, shipping, military sonars, fishing, and research activities. These disturbances affect the quality of data packet delivery in the underwater environment.

#### 2.1.4. Low Bandwidth

The operational frequency range of the underwater sensor nodes is primarily restricted due to the usage of acoustic waves as the medium of transmission. The bandwidth is a meager spectrum that lies between 1 kHz and 50 kHz. This poses a significant problem for routing protocols as it requires an enormous amount of data exchange at various stages like discovery and maintenance. Tight bandwidth constraints put challenging design constraints on acoustic systems. In order to perform communication with AUVs, it is more important to have a wider bandwidth rather than a rate. Moreover, the routing protocols are forced to choose routing paths from this small frequency range for data delivery. However, due to the dynamic nature of UASNs, continuous node mobility, communication voids, and limited battery storage often lead to degraded network performance. In this complicated underwater environment, how to route data packets promptly and effectively even with the presence of a communication void is the most challenging research question.

#### 2.1.5. Low Data Rate

Speed is a crucial factor when it comes to information exchange. The faster the data reaches the destination, the better. Unlike its counterpart (terrestrial environment), the speed at which data is transmitted in the underwater environment is influenced by numerous factors. Firstly, the propagation speed of acoustic waves is inferior to RF waves by many folds that create room for propagation delay. Secondly, there are various persuasive components like depth, temperature, and the degree of salinity of the water. The data rate is meager and accounts for approximately 100 kbps or occasionally a bit more.

#### 2.1.6. Transmission Loss

The hurdles when it comes to underwater sensor network implementation are numerous. Acoustic waves do not guarantee any reliability for the network. On top of that, path loss, Doppler spreading, and high latency will provide a clear picture that there is a considerable amount of packet loss. Transmission loss in any network is not a desirable outcome. Interference is one of the main reasons for packet loss to occur. When the same nodes participate in data transmission continuously for an extended period, the battery can run out, resulting in a communication blackout, and the node will no longer be able to transfer data collected from some places in the network. The acoustic signals have open channels, which are more likely to be utilized by an attacker or malware and to wreak havoc in critical services like routing, localization, and synchronization. Delay variance and bit error are two constituents that can lead to a high amount of packet loss and bit error rates.

#### 2.1.7. Error Prone

The underwater sensor nodes, unlike their conventional counterparts, are not reliable. The environment in which it has been implemented does not support its operation. The mobility, high latency, delay in propagation, high interference, noise, etc., make them highly susceptible to errors. The changes that manifest due to the variation in salinity, depth, and acoustic speed have an implicit effect on making the data transmission process error prone.

#### 2.1.8. High Energy Consumption

Energy drainage is a significant problem in UASNs. Communication between various nodes in a network rudimentarily requires the acknowledgment of its position. The nodes are constantly swaying in harmony with the ocean currents, and it is essential to update their position consistently with their neighbors for effective participation in the data transmission process. Ironically, this position-update process drains quite some energy from these sensor nodes. Another avenue wherein the power consumption rates rocket is when packets have to be retransmitted due to high interference. The data load bestowed on end nodes that connects to the surface stations rapidly depletes the battery power, resulting in the termination of connection with the rest of the nodes in the underwater network. The consumption rates vary with the depth in which it is implemented; the battery is expected to operate well in shallow and deep-water conditions.

#### 2.1.9. Channel Attenuation

Channel attenuation is another dilemma that underwater sensor nodes have to confront. The implementation of sensor nodes in the ocean bed is beneficial only if it can collect and transfer data, but due to channel attenuation, the data collected cannot be efficiently extracted from the received signal.

#### 2.1.10. Short Network Lifetime

The pivot grounds for the short lifetime of underwater sensor nodes are due to its source of energy, the battery storage. The nodes extensively consume energy while localization, routing, and data transfer. The hostile underwater condition makes the replacement of cells regularly a challenging task. Therefore, an efficient routing protocol has to consider energy consumption while making decisions on routing path selection. Furthermore, if the nodes run out of energy, it will result in the formation of dead nodes that can affect the network performance and data transmission to the surface stations.

#### 2.1.11. Security and Privacy Issues

UAWNs are made and deployed to monitor places consistently that are far from the shoreline. There is a high chance that the nodes are deployed in strategic waters for specific applications. Attackers can easily manipulate UASNs to inject malicious attacks upon the network. They can also be physically destroyed by enemy divers/AUVs. In the worst-case scenario, attackers can inject fake nodes into the network to provide misguided information and use compromised nodes to extract exclusive data from the network.

#### 2.1.12. Physical Challenges

The sensor nodes have to be fabricated so that they are compact, rigid, and waterproof and should also be able to withstand the pressure of water. Marine life is the next physical challenge that these sensor nodes have to face. In reality, it is physically impossible to protect every one of the nodes in the network.

### 2.2. Applications of UASNs

This section presents an overview of the major applications that use UASNs.

#### 2.2.1. Military Applications

The military applications of UWSNs can cover a wide range of requirements from monitoring to reconnaissance. In 1982, the United Nations Convention On the Law of the Sea allowed countries to exercise jurisdiction on territorial waters up to 200 nautical miles along the baseline. The naval force guards the coastline against invaders, but the underwater regions in strategically important areas are vulnerable. This vulnerability can be defeated with the help of UASNs. It will enable the militaries to detect enemy divers, submarines, torpedoes, AUVs, and naval mines. The ability to get real-time data will enhance strategic decision-making.

#### 2.2.2. Oceanography

Oceanography is the study of physical and biological aspects of the ocean. Oceanographic studies and researches will provide humans with the capability to understand the various phenomena that take place in the ocean and also be able to predict or artificially simulate similar conditions that will benefit human society. Oceanography can provide efficient analysis if it can collect real-time data. UASNs can be utilized to perform experiments to unravel the mysteries of the underwater world consistently, which will indirectly help us to obtain solutions to various problems oceanographic problems.

#### 2.2.3. Coral Conservation

Corals are one of the most beautiful living things on the planet. It takes millions of years to form barrier reefs. The Great Barrier Reef in Australia is the most extensive collection of corals on the phase of the Earth. However, it is dying due to coral bleaching due to the shift in climatic conditions throughout the world. Coral reefs around the globe are on the verge of extinction, and nations are trying to change the situation. Human interference has the likeliness to accelerate the degradation process, but data collection is seemingly impossible without human interference. UASNs are a profound solution that can provide real-time data to conservationists by limiting human interference.

#### 2.2.4. Resource Tapping

The Earth has resources that are tucked away in the depth of the ocean. UASNs provide a way to get the know-how of these varied resources. UASNs will enable us to find out the location, approximate quantity, and dispersion pattern of resources present in the ocean bed. Petroleum and natural gases are an inevitable part of our civilization, which are unfortunately limited. New potential sources can be located for extraction using UASNs.

#### 2.2.5. Fishing, Farming, and Recreation

The fishing industry will benefit from the use of UASNs as they will help locate groups of fish. Underwater farming has been used to cultivate seaweed, lettuce, basil, etc., in countries like Japan and Italy. Knowing the nature of the ocean is an integral part of taking out cruises for recreation purposes deep into the ocean. UASNs can tell leisure seekers about the risks of a tsunami or hurricane before they embark on a cruise.

#### 2.2.6. Disaster Prevention/Prediction

The implementation of UASNs will enable us to detect in advance any underwater earthquakes and volcanic eruptions, which will help us prevent or predict disasters. Many aircraft have gone missing over these years in oceans, and no data about their disappearance was harnessed. One of such shocking incidents is that of Malaysia Airlines 370. UASNs, provided it is implemented correctly, will enhance us to chart the ocean, and it is possible to derive a pinpoint location of any possible crash site.

#### 2.2.7. Climate Change

The rising sea levels and warmth have grabbed international attention. The polar ice caps are at the risk of meltdown. Accurate screening and reports of the polar meltdown can be undertaken with the help of UASNs, which will help researchers and environmentalists to find solutions to these baffling dilemmas.

## 3. Opportunistic Routing in UASNs

The uncertainty of the underwater environment poses many underlying threats to establishing efficient communication strategies. The constraints on power and the constant movement of nodes due to tides make opportunistic routing (OR) a viable solution. The opportunistic routing owns different modus operandi. On receiving a data packet, the host node takes into consideration a set of eligible neighboring nodes and prioritizes them based on various parameters. These parameters are different facets like the node closest to the destination and least power draining. A suitable packet forwarder gets opted from the candidate set based on priority and availability. Thus, in the case of unreliable underwater communication, OR proves to be promising as it provides extended reliability, robustness, and QoS than other legacy routing methods.

The principle of opportunistic routing idea was initially developed in ExOR [19] in 2005. The notable advantage of this protocol is that this protocol exploits the multiplex communication opportunities in which the broadcast character belonging to the wireless network develops. The fundamental working of opportunistic routing can be implemented in this protocol, and the three main steps include the following: Initially, the sender node can broadcast the message data. Secondly, upon receiving that data, one relay node is selected as the best forwarder node. After that, the selected best relay node transports the message transmission to the next best relay, and so on. The method is continued until the data reaches the target position. Compared to traditional routing methods, the next-hop relay is selected only after it has received the data, thereby reducing the number of data retransmissions.

The UASN's operation using acoustic channels for communication has many downfalls as there is a prevalence of solid attenuation, time-varying multipath, ambient noise, and modicum propagation speed. All of these contribute to increased delay, error, limited bandwidth, high energy consumption, communication cost, and at times temporary loss of connectivity among nodes of the network. The profound influence of channel fading is crucial to confront as it can directly impact declining routing performance. The scope of application of OR is of paramount importance because it has significantly low retransmission rates, in turn reducing the power consumption. Assured packet delivery facilitation by opportunistic routing ensures no wastage of network resources. It also reduces the chance of system collapse and diminishes retransmission costs. Additionally, opportunistic routing is a versatile choice as it applies to a variety of networks.

Opportunistic routing facilitates a dynamic and instant multiple-path routing technique through opportunistic relay selection, unlike the traditional routing method. Instead of a single precomputed relay, opportunistic routing initially broadcasts a data message to a set of forwarder relay nodes. Fundamentally, these forwarders are organized according to a particular unit. The idea of this method is to select the best forwarder relay among all the nodes. This selected relay manages the process of forwarding the packets. These steps are recursively executed until the packet is transmitted to the target destination. The rudimentary opportunistic routing mechanism consists of the following four steps:

- Forwarder relay set choosing
- Broadcasting of data to forwarder nodes
- Coordination scheme is used for best relay selection
- Forwarding of data by the best relay

Each node in opportunistic routing broadcasts a data packet to various adjacent hops periodically. Hence, if communication to one neighbor crashes, another nearby node that has received the data packet can transmit it. OR defines a group of various next hops as the best forwarder relay collection and indicates it as a forwarder relay set (FRS). When a message gets transmitted to FRS, numerous forwarders can obtain a similar message packet. We can avoid duplicate transmission by selecting a single candidate as the best relay. Each node in the FRS is allocated a priority that is calculated based on a predefined variable. Suppose the node with the most significant priority present in the FRS favorably acquires the message, it transmits that to the target. Otherwise, the node that has the next most significant priority transmits the data packet, and so forth. The leftover candidates will discard this data packet. The FRS selection is divided into three main components as follows: (a) forwarder relay discovery, (b) prioritization variable calculation, and (c) forwarder relays selection, prioritization, and filtering.

To find out the neighbor node, periodic or nonperiodic packets are broadcasted. This neighbor node depends on the link quality, which is changeable as well as dynamic. Hence, this phase is given the charge of computing the stability and quality of the links to reach the neighborhood. Based on these values, a group of nodes is determined. Initially, every node located in the vicinity of the sender node is added to the FRS. Then, the forwarders are taken and sorted based on the chosen variable. After an FRS is elected, priorities are given to forwarder relays based on a specific value. So, the variable selection affects the network throughput significantly. The priority variable election depends on the routing application needs and targets. For some applications, such as emergency recovery, the position data is essential. Consequently, the relay nodes must know their location, and routing can be executed by selecting the relay that is locationally nearest to the target node. Controlling the number of forwarder relays can reduce the overhead and duplicate data transmissions. Moreover, since the size of FRS grows, the number of forwarders who cannot listen to one another also increases. This leads to duplicate packet transmissions. Hence, it is suitable to avoid some forwarder candidates from the FRS. This approach is termed candidate filtering or forwarder. The conventionally used filtering method avoids the forwarders, which are not suited instead of the source. But somehow, this policy cannot guarantee efficient network performance. Another method of FRS creation is discussed in some previous works. The technique is based on implementing an algorithm that can optimize correctly and compute the optimal forwarder relays set for every node, such as forwarder relay sets that are created by Dijkstra's algorithm. However, these methods do not solve the issues of duplicate data transmission.

The optimal relay selection that uses a coordination scheme is used for the coordination of packet forwarding operation between next near nodes. This scheme is responsible for selecting the most suitable forwarder relay to push forward the data packet. Coordination methods need signaling between forwarders. The basic coordination schemes are generally classified into a timer-based, contention-based method, and token-based coordination scheme. In a contention-based method, the main principle is that forwarder relays contend to transmit the data packet with the help of control messages. For example, if a sender node transmits a forward request, its near hop nodes have to compete with themselves to come to a consensus on the forwarding of the data packets. In the timer coordination method, the forwarder relays are supposed to be ranked according to a specific priority value. This rank is commonly added with the message header, which is consistent with the hierarchy in which potential forwarders are permitted to respond. Thus, the largest priority node is allowed to respond to the first slot. The next priority node responds to the upcoming time slot, etc. However, this method is straightforward and easy to carry out, timer-based coordination that incurs some delay, affecting network performance. Another method is the token-based coordination scheme, in which the transferring of data packets is only possible through a token holder. In this scheme, the duplicate message transmission is completely prevented, but it faces increased overhead control. A forwarder (relay) node contains the overhead data packets that are being sent when a token arrives. Tokens travel with connected forwarders because more miniature priority forwarder relays can listen to large priority nodes. If no token arrives, the candidates may be moved into an idle state, slowing down the network.

## 4. Location-Based Opportunistic Routing Protocols in UWSNs

All routing protocols for UAWNs can be classified as location-based protocols and location-free protocols. The location-based protocols instruments data contained within sensor nodes that are mainly two/three-dimensional position coordinates. At the same time, the location-free protocols/depth-based protocols depend on the information related to pressure on sensor nodes. The focus of this study lies in location-based protocols as they provide better performance than location-free protocols. Vector-based forwarding (VBF) [21] was one of the earliest protocols proposed in this category. This protocol can fabricate some virtual vector pipe that exists between the source and the destination. Only the nodes in the vicinity of the “vector” right through the source and destination will have the ability to do message forwarding. Hence, routing involves only a tiny group of nodes.

Similarly, numerous location-based protocols were proposed for UASNs. Some of the protocols focused on improving energy efficiency, while others focused on improving QoS parameters like delay and delivery ratio. Recently, many hybrid protocols also have been proposed which consider both energy efficiency and QoS. This section presents a comprehensive discussion on all the latest location-based protocols proposed for UASNs.

VBF makes use of the node location information to make the routing decisions. The knowledge of the position of nodes encourages it to be faster, reliable, and scalable. With the protocol, a virtualized pipe is created from source to destination, and those nodes in the pipe possess a higher probability of becoming the forwarder nodes, while the nodes outside are disregarded. Sink-initiated query and source-initiated query are the two main ways in which VBF addresses routes to different queries. Conceptually, all nodes inside the virtual pipe have the eligibility to forward the packets, but due to limitations like energy, mobility, and propagation delay of acoustic waves, a self-adaptation algorithm was suggested. Another protocol, directional flooding-based routing (DFR) [22] defines a forwarding method formulated by the angle among the center and intermediate nodes. The nodes are responsible for forwarding the data packets through a flooding method. It also considers the quality of the link between the sender and the destination node. A significant concern with this protocol is redundant data transmission and increased energy consumption. The information-carrying routing protocol (ICRP) [23] is an influential conservative, continuous, and versatile directing protocol. The sender hub checks the current location to the final destination when it owns the data to be sent. If there is no current course or path, it starts a path development process by communicating with the information packet, conveying the route disclosure message. Every node present on the network communicates to maintain the reverse route with the information path.

Hop-by-hop vector-based forwarding (HH-VBF) [24] is another variation of VBF where each forwarder resorts to a different routing vector. HH-VBF rudimentarily is just a version of the vector-based forwarding protocol. HH-VBF is a viable option compared to VBF as it can work well with sparse networks and is not liable to the routing pipe radius threshold. However, there is an increase in the computational delay, which in turn degrades the network performance. Reliable and energy balanced routing (REBAR) protocol [25] is a routing protocol that is energy efficient that helps in varying the broadcast domain. REBAR has good reliability and increased lifespan of the network. To balance the energy consumption in the network, a flexible scheme is developed to establish the data propagation range. Here, the nodes near the destination have a modicum radius. However, the increased node movements may expend an excessive amount of energy, resulting in degradation of performance. Vector-based void avoidance (VBVA) [26] protocol is simply an extension of the VBF protocol and focuses on addressing the void problem and energy efficiency in UASNs. The protocol works similarly to VBF when there is no void but uses a revised strategy when voids appear in the network. This helps the protocol to maintain better energy efficiency even with voids in the network.

The energy-efficient and collision aware (EECA) [27] multiple-path routing methods are founded on computing two different collision-free paths using restricted-energy modified flooding. It is one of the earliest protocols that gave equal importance to the betterment of QoS and energy efficiency in the network. Here, multipath power-control transmission (MPT) allows packet data transfer within limited end-to-end data error value and reduced power of transmission. The reliable energy-efficient routing protocol [28] functions on the foundation of link quality, physical data distance, and energy available in the UASN. These three values are calculated and shared with all nodes in the network. The protocol uses a local flooding mechanism with an adaptive selection and gives good reliability and energy efficiency performance.

Location-aware routing protocol (LARP) [29], the GPS is used to identify the exact area of the sink nodes. The sink nodes then broadcast the location information in the network. At the least three sink nodes are used for reference, other nodes in the network calculate their position. The sender can locate the next hop by broadcasting two things as follows: (1) location of the destination node and (2) moving direction of the packet. Packets are forwarded if the receiving node discovers that it is moving in a similar direction. The quality-of-service aware directional flooding-based routing (QoSDFR) [30] extends the DFR protocol. In this routing strategy, the sink node is responsible for sending feedback to various other nodes in the network about the channel condition, and based on the feedback, the optimal forwarder is selected. Protocol results in high throughput because of the limited energy consumption and varying channel conditions.

Scalable and efficient data gathering (SEDG) [31] protocol tries to increase the delivery ratio of the packet and also saves the modicum energy by feasible assignment of the member nodes and gateway node (GN). Here, an autonomous underwater vehicle (AUV) goes through the network area with a precomputed elliptical route and collects data from the gateway node (GN). AUV-aided efficient data gathering (AEDG) routing protocol [32] employs an AUV to gather information from gateways or intermediate nodes and use the shortest path tree (SPT) algorithm to balance the energy consumption. Besides that, AEGD designs a model that improves the result and saves energy by reducing the node members. Furthermore, the nodes live for an extended time to transfer data, thereby increasing delivery chances. The delay-aware energy-efficient routing protocol (DEEP) [33] is a delay-aware routing protocol dependent on collision rate and energy. DEEP makes use of an adaptable node aimed to minimize the collision rate. All the intermediate nodes are elected by virtue of delivery ratio and link quality. In the channel aware routing protocol (CARP) [34], the next-hop transmitter node is elected due to its distance from the previous intermediate node and available energy. Here, every intermediate node is familiar with its neighborhood between the destination node and the next hop. Sender then broadcasts a PING message to the network to compute the next forwarder. Considering a case where the hop value of a sink is lower than the sender node, it replies a PONG data. CARP uses an efficient relay selection method, which doubles the packet delivery ratio.

The novel efficiency forwarding protocol (NEFP) [35] is a proactive anycast routing protocol proposed for UWSNs. It promotes three different approaches. One defines a routing method that avoids unnecessary forwarding of packets where the collision dilemma is averted using a timer. Moreover, finally, the design uses Markov chains to calculate the probability of forwarding the data packets that encourages adaptability to constantly changing network topology. Nevertheless, the performance of the suggested protocol is decreased in the sparse region and as a result, reduces the number of forwards in the phases. Geographic and opportunistic routing protocol with depth adjustment (GEDAR) [36] is a geo-opportunistic routing protocol proposed for a minute-monitoring task. It utilizes a greedy forwarding method to advance the message towards the next hop. The source node chooses the best candidate from the forwarding set. The opportunistic routing in GEDAR reduces the number of retransmissions. GEDAR uses a recovery mode that helps to avoid the void areas. If a node is present in the void area, it will adjust its depth to overcome the void, and new messages will be queued. The greedy strategy will reschedule the node later. Markov model-based routing (MMVR) [37] selects its route from the lower surface to the top level based on changing data traffic. The routes are stable and adaptable, with fewer hops from the sender node and destination. In a localization-based dynamic routing protocol (LBDR) [38], the network is split into smaller layers, and a virtual routing vector is made within the sub-layers. Nodes will move in and out of the virtual vector based on the water current, resulting in high throughput. Void handling geo-opportunistic routing (VHGOR) [39] protocol focuses more on efficiently handling the communication holes in the network. Here, a quick hull algorithm is used to avoid a convex hull. When the node or hub reaches a convex region, rebuilding the convex void helps check an alternate and different way to resume the greedy transmission. VHGOR improves the network performance in networks with voids compared to other routing protocols.

Geographic and opportunistic routing (GOR) [40] protocol shows efficient multi-hop data transmission in UWSNs with an upgraded strategy compared to previous protocols. Sometimes, this method gives room for the formation of the void region, and GOR tackles this issue using some void-handling algorithms. The framework considers network density, traffic load, and energy control features to bypass the empty region. The range-based low overhead localization technique (LOTUS) [41] significantly improves on earlier versions of the localization protocols. The protocol can estimate locations based on only two references, enabling this technique to work in networks with fewer nodes. The geographical duplicate reduction flooding (GDflood) [42] considers the location data regarding sensor nodes and joins it with network coding. Energy-efficient grid routing based on 3D cubes (EGRCs) [43] employs a 3D cube network that is subdivided into small cubic clusters. The cluster head is determined based on the remaining energy and position of the intermediate node. All the cluster heads then compute their intermediate node based upon the delay and location. EGRCs reduce energy consumption and end-to-end delay and increase the network performance.

Mobile energy-efficient square routing (MEES) [44] is a routing protocol focusing on energy efficiency in underwater sensor networks. The method uses a division of the network field into dense and sparse regions. A major advantage of this method is that, the mobile sink shifts in a clockwise direction that ensures the highest coverage of nodes in the network which will, in turn, result in high throughput and energy consumption. Topology control vector-based forwarding (TC-VBF) [45] is a revamped version of VBF, which tries to address the limitation of VBF in light conditions. Another protocol energy-efficient multipath grid-based geographic routing protocol (EMGGR) [46] fragments the network into 3D grids. The routing is executed in a grid-by-grid fashion with the help of gateway nodes. Disjoint paths result in high energy efficiency and a good packet delivery ratio. Balanced multiobjective optimized opportunistic routing (BMOOR) protocol [47] uses a strategy where the data from the lower surface takes the best route through the intermediate nodes to the top-level sink. Here, the nodes are located as per dynamic assessment with regards to optimal energy forwarders. The BMOOR protocol needs no spatial data, which is costly in UWSN. The protocol is developed using a generation-based bio-inspired, meta-heuristic algorithm. This helps in delay depreciation and maximization of delivery ratio, and thereby the network lifetime is enhanced. Another proposed protocol for UWSN is energy-efficient interference aware routing (EEIAR) [48] that opts for the best forwarder following the shortest distance. The shortest distance determination decreases the propagation delay. The power control-based sharp directing routing (PCR) [49] selects the most optimal transmission power level available at each submerged sensor node, which helps improve the packet delivery conveyance at each round. Also, it condemns the usage of high-power transmission and the uncontrolled consideration of neighboring hubs in the following hop candidate set, which would end up being the root cause for building the energy utilization on the network. The simulation outcomes depict that PCR diminishes the energy expenditure by adjusting the transmission power and electing the best candidates. The stateless opportunistic routing protocol (SORP) [50]uses a novel method to employ a variable forwarding area that can be reshaped and replaced according to the regional density and placement of the potential forwarding nodes to improve the energy and reliability. The protocol gives good performance compared to the previous protocols. Glider-assisted link disruption restoration mechanism (GALDRM) [51] uses a link disordering recognition with a related link rebuilding method. In the connection acknowledgment system, the group nodes gather the link data. The cluster heads gather the disruption data in link disruption and then schedules gliders as relay nodes to revive the link. Utility capacity is built up by limiting the channel. A multiplier technique illuminates the ideal area of a lightweight flyer. The simulation outputs exhibit a glider-assisted reconditioning procedure that helps to reduce energy consumption. The energy-aware void-avoidable routing protocol (EAVARP) [52] expands the network lifetime and packet delivery rate in underwater sensor networks. EAVARP includes layering and data collection phase with the help of directional forwarding strategy and uses residual energy and data transmission to avoid cyclic transmission and flooding. Fuzzy logic-based VBF protocol (FVBF) [53] improves VBF protocol. It focuses more on the selection of a single forwarder node in VBF. FVBF is the fuzzy logic-based VBF protocol. The best forwarding node is chosen according to the angle of projection distance and the battery level. The smallest distance shows that the node is in the vicinity of the target node. The projection angle allows it to be selected onto the virtual routing vector pipe. The best advantage of this protocol is that it achieves better energy and throughput. However, nodes in the selected vector terminate on dealing with a high load of the message, which is similar to the conditions in VBF.

Mobility-assisted geo-opportunistic routing (MSAGOR) [54] protocol is mainly based on interference avoidance. Here, the network region is fragmented into compact cubes to diminish the interference, which helps to make additional well-informed routing strategies for better energy utilization. Moreover, an optimal number of transmitting nodes are selected from each cube based on its distance to the destination. This proximity will help to avoid void nodes. The extensive simulation results reveal that this protocol will maximize the delivery ratio and network lifetime. Totally, opportunistic routing algorithm (TORA) [55] is an anycast, geographic opportunistic routing protocol proposed for UWSN. The protocol is implemented to avert parallel transmission, bring down end-to-end delay in the network, tame the dilemma of void regions, and enhance network throughput. TORA uses time on arrival and its range-based equation to localize nodes. The energy-aware opportunistic routing (EnOR) [56] is an energy-aware opportunistic routing (EnOR) protocol that can adjust the priority level of forwarding between candidate nodes. This leads to steady energy utilization and increased network lifetime. By using the residual energy, link reliability, packet advancement ratio, and EnOR change the priority of transmission level. Adaptive hop-by-hop cone vector-based forwarding protocol [57] tries to improve the reliability of data transmissions in the sparse sensor regions by making some modifications to the base angle of the cone as per the network structure. These protocols improve the network performance by reducing the number of duplicate packets and also enable a better selection of the potential forwarder node.

Authors in reference [58] discuss implementing a modified strategy for depth-based routing that can transfer the data reliably to the surface sonobuoy. The technique mainly uses the 2-hop neighbor technique and tries to improve the delivery ratio of packets in the network. Authors in reference [59] proposed a technique combining the ant colony optimization algorithm, artificial fish swarm algorithm, and dynamic coded cooperation to improve efficiency by reducing energy consumption. Improving the flexibility of the protocol with the network was one of the major tasks of the proposed algorithm, along with finding the most optimal route. In reference [60], authors presented a Q-learning-based multi-hop cooperative routing protocol for underwater networks. Using this algorithm, the nodes with maximum *Q*-value were selected as the next forwarders in the network to transfer data from the source to the destination. A coding-aware strategy was proposed for efficient routing in networks with the sparse deployment of nodes [61]. The topological information was used to expand the candidate set using the protocol. An interesting approach that utilizes AUVs to carry sensor nodes to repair the routing voids when foreseeing the occurrence of voids was proposed in reference [62]. The protocol initially predicted the location for repair and then directed the AUVs to the particular location to carry out the repair process. Most of the proposed protocols are complex and incur high overhead, which degrades the performance of the network. Although many of the current protocols improve the data delivery ratio significantly, it comes at the cost of increased energy consumption. It is vital to develop a simple to implement a protocol that can take care of energy efficiency in the network while ensuring reduced delay in the network.

## 5. Energy-Efficient Location-Based Opportunistic Routing Protocol (EELORP)

In this section, we present the discussion on the proposed energy-efficient location-based opportunistic routing protocol (EELORP) that is designed to provide better energy efficiency and data delivery with minimum delay.

### 5.1. Theoretical Analysis

Initially, we try to provide a theoretical analysis to the proposed protocol. The focus is mainly on the delay of transmissions that can be reduced further to enhance the performance of the system. In the underwater network, a delay occurs within two different links, the wireless sensor to the wireless controller and wireless controller to the actuators. The delays are denoted by *T*_*w*(*s* − *c*)_ and *T*_*w*(*c* − *a*)_. Assuming the controller to be time invariant, the delays due to two sources are combined together to get total wireless sensor network delay as follows:

(1) $$\begin{array}{c} \mathrm{Twt}=\mathrm{Tw}\left(s-c\right)+\mathrm{Tw}\left(c-a\right)\text{.} \end{array}$$

The computation delay of the controller can also be included in the total wireless sensor network delay. As the assumption in the wireless controller is time invariant, the decision of controller *d*_(*t*)_ is independent of the time it receives the sample *S* ((*γb*). So, the total wireless sensor network delay is only important for us. The analysis of UWSN stability is carried out by assuming two different scenarios as follows: (a) the continuous UWSN network delay system is considered by determining UWSN stability with constant network delay and (b) the discrete UWSN network delay system is considered by determining UWSN stability with time-varying networking delay.

For a continuous UWSN network-delayed system, the UWSN having total network delay as *T*_*WT*_ at the time *t* = ɤ*b* is considered. The assumption is extended by making *T*_*wt*_ < *b* for all values of “ɤ” belonging to “*S*” with ɤ ∈ *s*. The system is modeled mathematically as follows:

(2) $$\begin{array}{c} \frac{\partial }{\partial t}l\left(t\right)=Pl\left(t\right)+Qd\left(t-T_{\text{WT}}\right), \end{array}$$

where “*t*” belongs to [*γb*,  *γb*+*b*]. Also with *P*, *Q*, *R*, and *S* as known matrices, we have the following relation:

(3) $$\begin{array}{c} M\left(t\right)=R\gamma \left(t\right)+Sd\left(t\right). \end{array}$$

*d* (*t*) is the received signal with no delay and *d*(*t* − *T*_WT_) is the received signal with delay. In the case of *d* (*t*), that is, received signal with no delay *d*(*t*)  =  *d*(*γb*) for *t*  ∈ [*γb*, (*γb*+*b*)].

**Proposition 1 .**

The UWSN with the delay mentioned above validates the below-mentioned difference equations. The derived equation is as follows:

(4) $$\begin{array}{c} l\left(\gamma b+b\right)=\tau l\left(\gamma b\right)+\varepsilon_{0}\left(T_{\text{WT}}\right)d\left(\gamma b\right)+\varepsilon_{1}\left(T_{\text{WT}}\right)\left(d\left(\gamma b-b\right)\right). \end{array}$$

For *τ*=∫_0_^*b*^*e*^*Pb*^ , we obtain the following equation:

(5) $$\begin{array}{c} \varepsilon_{0}\left(T_{\text{WT}}\right)=\;\int_{0}^{b-T_{\text{WT}}}e^{Pb}d\gamma \varphi ,\\ \varepsilon_{1}\left(T_{\text{WT}}\right)=\int_{b-T_{\text{WT}}}^{b}e^{Pb}d\gamma \varphi . \end{array}$$

Now, we have the following equation:

(6) $$\begin{array}{c} l\left(t\right)=e^{P_{\left(t\right)}}+\int_{0}^{t}P\left(t-r\right)\varphi \text{d}\left(\gamma \right)\text{d}\gamma . \end{array}$$

If the delay *t*_0_ > 0, then the above equation is rewritten as follows:

(7) $$\begin{array}{c} l\left(t\right)=e^{P_{\left(t-t_{0}\right)}}l\left(t_{0}\right)+\int_{t_{0}}^{t}P\left(t-r\right)\varphi \text{d}\left(\gamma \right)\text{d}\gamma . \end{array}$$

For for *t* > *t*_0_, we have the following equation:

(8) $$\begin{array}{c} l\left(\gamma b+b\right)=\tau l\left(\gamma b\right)+\in d\left(\gamma b\right), \end{array}$$

where *τ*= *e*^*Pb*^  and. *ε*=∫_0_^*b*^*e*^*Pr*^ *dγ*  *φ*.

Applying equation (7) to (4), we obtain the following equation:

(9) $$\begin{array}{c} l\left(\right)\left(\left(\gamma b+b\right)\right)=e^{Pb}l\;\left(\gamma b\right)+\;\int_{\gamma b}^{\gamma b+b}e^{P\left(\gamma b+b-\;\gamma \right)}\text{d}\gamma \varphi \text{d}\left(rb-T_{\text{WT}}\right)\text{d}\gamma ,\\ =\tau l\left(\gamma b\right)+\;\int_{\gamma b}^{\gamma b+T_{\text{WT}}}e^{P\left(\gamma b+b-\;\gamma \right)}\text{d}\gamma \varphi \text{d}\left(rb-b\right)+\int_{\gamma b+T_{\text{WT}}}^{\gamma b+b}e^{P\left(\gamma b+b-\;\gamma \right)}\text{d}\gamma \varphi \text{d}\left(rb\right),\\ \gamma^{1\;}=\;\left(\gamma b+b-\;\gamma \right),\\ \tau l\left(\gamma b\right)-\;\int_{b}^{b+T_{\text{WT}}}e^{P\gamma^{1}}\text{d}\gamma^{1}\varphi \text{d}\left(\gamma b-b\right)-\int_{b-T_{\text{WT}}}^{0}e^{P\gamma^{1}}\text{d}\gamma^{1}\varphi \text{d}\left(\gamma^{1}b\right),\\ =\;\tau l\left(\gamma b\right)+\varepsilon_{0}\left(T_{\text{WT}}d\left(rb\right)\right)+\varepsilon_{1}\left(T_{\text{WT}}d\left(rb-b\right)\right). \end{array}$$

In other scenarios, multiple copies of the signal are transmitted in the time interval and they take different routes while travelling corresponding to the direct path and scattered path. The spread in the delay indicated as *σ*_*τ*_ of 1 to 3 .... *h*(*τ*) is the delay profile. Taking the Fourier transform, we obtain *H*(*f*)=∫_0_^∝^*h*(*τ*)*e*^−*J*2*πfτ* ^d*τ* . The coherence bandwidth at which the delay profile response is almost flat, if the signal bandwidth *β*_*s*_ <  *β*_*c*_ is less than coherence of *β*_*c* _=1/2*σ*_*τ*_.

Figure 2 shows the signal for *σ*_*τ*_ ≪ *T*_*s*_ or *σ*_*τ*_ ≫ *T*_signals_. So, the sound signal interferes each other significantly and so on as delay spread increases to *σ*_*τ*_ > *T*_signals_ and 1/*T*_signals_ > 1/*σ*_*τ*_, which implies to *β*_*s*_ > 2*β*_*c*_ obtained as the interference. The *T*_*x*_ is stable and *R*_*x*_ is moving towards *T*_*x*_, indicating the change in the frequency of sound varying due to relative motion between the *T*_*x*_ and *R*_*x*._

### 5.2. Simulation Results

In this section, we discuss the performance comparison of the proposed EELORP protocol by conducting simulations in Aqua-Sim [63–66]. Aqua-Sim is an extended version of NS-2 and offers easy implementation of underwater network scenarios. The parameters used for setting up the network are given in Table 2.

Using the simulations, we measure the energy consumption in nodes and the delay that occurred in the transmission of data in the UWSN. We also compare the results obtained by our proposed work with vector-based forwarding (VBF).  Figure 3 shows the energy consumption by nodes in the network. From the results obtained, we can see that the nodes consume less energy using the proposed EELORP protocol compared to VBF protocol. Initially, the nodes have the same level of energy consumption with both the protocols, but as the number of nodes increases, the energy consumption using VBF becomes more compared to the proposed scheme. This signifies the better energy efficiency offered by the proposed protocol.

Figure 4 shows the delay incurred in transmission of the data packets using the protocols in the UWSN. From the results, we can see that using the proposed method EELORP and VBF, the delay incurred remains almost similar when the number of nodes is less. But as the number of nodes increases, the EELORP has less delay compared to VBF in the network. Thus, our results show that the proposed protocol can be used efficiently for numerous possibilities in underwater acoustic sensor networks with reduced delay.

## 6. Future Research Directions

### 6.1. Energy Efficiency

This has emerged as one of the major research areas for opportunistic routing protocols in underwater acoustic sensor networks. With restrictions and various limitations in recharging the sensor nodes, it is very important for any routing protocol to minimize the energy usage in the nodes while ensuring that the data gets delivered to the destination. Numerous protocols have tried to improve the energy efficiency in the network, but as UASN has an unpredictable nature, we should for further improvement in this research direction.

### 6.2. Channel Utilization

The unique features of UASNs like high propagation delay, constant mobility of sensor nodes, high error rate, and interference lead to a major challenge in ensuring the efficient utilization of the channel. Most of the existing protocols have various limitations in channel utilization and this area would be a major area of focus.

### 6.3. Communication Holes

Dealing with communication holes is a major challenge in UASNs, especially in networks with sparse deployment. Frequent movement of the sensor nodes due to currents and other reasons and failure of sensor nodes due to energy drainage or damage create void areas in the network. Thus, nodes will be unable to find suitable neighbor nodes to forward the data packet to the destination.

### 6.4. Security

Security of the data transmitted has become one of the major requirements of the applications deploying UASNs. It is therefore vital for all the routing protocols to include a security mechanism that can secure the data from any attackers.

### 6.5. Reliable Delivery

Reliable delivery of data packet at the destination is a major challenge in UASNs with a dynamic environment. Due to multiple reasons like damage of nodes, lack of energy, voids, etc., the data packet might get lost in the network. It is very important for any protocol to have strategies to manage any data loss and to make sure that the data reaches the destination, also keeping the number of retransmissions to a minimum to save the energy of nodes.

## 7. Conclusion

This study presented a systematic survey on the location-based opportunistic routing protocols in underwater acoustic sensor networks. The study initially discussed the working of underwater sensor networks, the challenges and issues, the latest applications using UASNs, and the working of opportunistic routing in underwater acoustic sensor networks. A detailed discussion on all recently proposed location-based opportunistic routing protocols was presented with a focus on their design and working. A discussion on the design and working of an easy-to-implement energy-efficient location-based opportunistic routing protocol (EELORP) that can be used efficiently for numerous possibilities in underwater acoustic sensor networks with reduced delay was presented. A discussion on results obtained with simulations was then presented along with comparisons with existing protocols. Finally, a brief discussion on the future research directions was presented.

## Figures and Tables

**Figure 1:** Underwater acoustic sensor networks (UASNs).

**Figure 2:** Physical layer-related losses and interference.

**Figure 3:** Normalized energy consumption versus the number of nodes.

**Figure 4:** Delay versus number of nodes.

**Table 1:** Differences between the TWSN and UASN.

	TWSN	UASN
Mobility	Low/medium	High
Reliability	High	Low
Data rate	High	Low
Bandwidth	High	Low
Interference	Low	High
Propagation delay	Low	High
Energy usage	Low	High

**Table 2:** Simulation specifications.

Parameter name	Values
Simulator name	NS 2.35 with aqua-sim
Dimension of topology	1500 × 1500 × 1500 m
Transmission range	250 m
Antenna type	Omni-directional
Data rate	50 kbps
Packet size	25 to 125 bytes
Number of nodes	100 to 300
Simulation time	200 s
Number of simulation runs	10
Protocols	EELOP, VBF

## Data Availability

All the output data with details can be accessed through the first author at reasonable request (email: varunmenon@ieee.org).
